# Contribution of Adiponectin/Carnitine Palmityl Transferase 1A-Mediated Fatty Acid Metabolism during the Development of Idiopathic Pulmonary Fibrosis

**DOI:** 10.1155/2022/5265616

**Published:** 2022-08-17

**Authors:** Wenjuan Wu, Guojun Zhang, Lingxiao Qiu, Xueya Liu, Shuai Zhou, Jizhen Wu

**Affiliations:** ^1^Department of Geriatrics, Henan Provincial People's Hospital, The Affiliated People's Hospital of Zhengzhou University, Zhengzhou 450052, China; ^2^Department of Respiratory Medicine, The First Affiliated Hospital of Zhengzhou University, Zhengzhou 450052, China

## Abstract

Idiopathic pulmonary fibrosis (IPF) is a chronic progressive interstitial lung disease that leads rapidly to death. The present study is aimed at discovering the in-depth pathogenesis of IPF, exploring the role of adiponectin/carnitine palmityl transferase 1A- (APN/CPT1A-) mediated fatty acid metabolism during the development of IPF, and excavating its potential mechanism. Here, THP-1 cells were differentiated into M0 macrophages, followed by polarization to M1 macrophages upon hypoxia. Subsequently, lung fibroblast HFL-1 cells were stimulated by M1 macrophages to simulate hypoxia-related IPF condition *in vitro*. It was discovered that the stimulation of M1 macrophages promoted fibroblast proliferation and fibrosis formation *in vitro*, accompanied with a disorder of the APN/CPT1A pathway, an overproduction of lipid peroxides, and a low level of autophagy in HFL-1 cells. Thereafter, APN treatment or CPT1A overexpression greatly suppressed above lipid peroxide accumulation, fibroblast proliferation, and fibrosis but activated autophagy *in vitro*. Furthermore, an *in vivo* IPF rat model was established by injection of bleomycin (BLM). Consistently, CPT1A overexpression exerted a protective role against pulmonary fibrosis in vivo; however, the antifibrosis property of CPT1A was partly abolished by 3-methyladenine (an autophagy inhibitor). In summary, APN/CPT1A-mediated fatty acid metabolism exerted its protective role in IPF partly through activating autophagy, shedding a new prospective for the treatment of IPF.

## 1. Introduction

Idiopathic pulmonary fibrosis (IPF) is a chronic and irreversibly progressive lung disease characterized by abnormal fibroblast proliferation and extracellular matrix deposition along with inflammatory response and tissue structure destruction [1]. Nintedanib and pirfenidone are approved by FDA as the clinical drugs for IPF treatment, but they can only slow down the development of IPF, hardly to cure it; thus, patients with IPF invariably have a poor clinical outcome [2]. Numerous risk factors, such as inhalation, infection, and radiation, have been reported to contribute to IPF; however, the exact etiology and pathophysiological mechanisms involved in IPF still remain elusive [3]. Hypoxia is an important microenvironment factor in the progression of tissue fibrosis. In pulmonary fibrosis, the alveoli are replaced by fibrotic cells, suppressing oxygen exchange and leading to widespread hypoxia, which subsequently triggers continuous production of fibrogenic cytokines, excessive fibroblast proliferation, and perpetuation of late lung tissue injury [1, 4, 5]. The hypoxia-inducible factor (HIF), a transcription factor existing as a heterodimer composed of an *α*-subunit and a *β*-subunit, is a main mediator of the cellular response to hypoxia [6]. In particular, HIF-1*α* has been uncovered to be highly expressed in alveolar epithelial cells of patients with IPF, and HIF-1*α* acts as a prominent trigger factor contributing to the development of IPF [7, 8].

Autophagy is a conserved catabolic process to recycle cytosolic proteins and organelles through the lysosome-mediated degradation pathway. It is a dynamic process involved in various cellular processes, so as to maintain cellular homeostasis [9]. Autophagy serves as a pivotal role in the pathogenesis of tissue fibrosis, including renal fibrosis, liver fibrosis, and pulmonary fibrosis [2, 10, 11]. A reduced autophagy level in lung tissues of IPF patients has been demonstrated by researches [12, 13]. Macrophages, the first line of defense against the external stimuli, act as a crucial role in the pathogenesis of pulmonary fibrosis. Macrophages can be differentiated into two distinct subpopulations, namely, as classically activated proinflammatory M1 phenotype and alternatively activated (M2) phenotype accounting for anti-inflammation and tissue repair [14]. Tissue hypoxia can polarize macrophages through stabilizing HIF-1*α*, which has been reported to exhibit activating effects on macrophages and initiate inflammatory response [15]. Meanwhile, HIF-1*α* was also found to mediate autophagy in multiple fibrosis processes [10, 16]. Yet, the concrete association and molecular mechanism behind these observations in IPF have not been well-understood.

Adiponectin (APN, also named as Adipo Q, ACRP30, and gelatin-binding protein-28), a specific adipocytokine predominantly secreted by adipocytes, has gained much attention in the last decade attributed to its physiologically regulatory functions in humans and rodents [17]. The effects of APN are mediated by APN receptors, which occur as two isoforms (AdipoR1 and AdipoR2). It has been revealed that APN reduces the intracellular lipid content through two approaches: one is to indirectly regulate fatty acid oxidation via the insulin/insulin-like growth factor (IGF) system and the other is to directly stimulate fatty acid oxidation and reduce fatty acid synthesis via activating 5′-AMP-activated protein kinase (AMPK)/carnitine palmityl transferase 1 (CPT1) [18–20]. The CPT1 family, comprising CPT1A, CPT1B, and CPT1C, is the key enzyme of fatty acid metabolism [21]. Deranged fatty acid composition or abnormal fatty acid metabolism is critical to contribute to pulmonary fibrosis [22–24]. In addition, the recent evidence uncovers the potential role of APN against multiple fibrotic diseases, including liver, cardiac, and pulmonary fibrosis [25–27]. A dysregulated CPT1A activity was discovered in lung macrophages from IPF patients, indicating a critical role of CPT1A in pulmonary fibrosis [28]. Thus, whether APN/CPT1A-mediated fatty acid metabolism exerts effects during the process attracted our attention. Of note, hypoxia caused a low expression of APN, while APN could activate macrophage autophagy to protect against cardiac fibrosis [29, 30]. Hence, whether APN/CPT1A-mediated fatty acid metabolism is involved in hypoxia-induced pulmonary fibrosis also deserves to be explored.

Based on the findings above, we aim to explore the critical role of APN/CPT1A in pulmonary fibrosis and to make an in-depth research on the regulatory mechanism underlying hypoxia-mediated pulmonary fibrosis.

## 2. Materials and Methods

### 2.1. Cell Culture and Treatment

Human monocytic leukemia THP-1 cells (TIB-202) and human lung fibroblast cells (HFL-1; CCL-153) were obtained from the American Type Culture Collection (ATCC; USA). THP-1 cells were cultured in RPMI-1640 medium (Gibco, Thermo Fisher Scientific, USA) supplemented with 10% fetal bovine serum (FBS; Gibco), whereas HFL-1 cells were cultured in F-12K medium (Invitrogen, USA) containing 10% FBS. Cells were maintained at 37°C and 5% CO_2_ in a humidified incubator.

THP-1 cells were treated with 150 ng/ml phorbol 12-myristate 13-acetate (PMA; P8139, Sigma-Aldrich, USA) for 24 h to obtain macrophage-like M0 cells [31], followed by exposure to hypoxia (atmosphere of 5% CO_2_ and 95% N_2_).

For cocultivation, a transwell (Corning, USA) coculture system was employed as described previously [32, 33]. Briefly, the differentiated M0 macrophages and the polarized M1 macrophages as described above were seeded in the upper chamber, and the HFL-1 cells were plated into the bottom chamber for cocultivation for 48 h.

### 2.2. Cell Transfection

The full length of the CPT1A open reading frame was amplified and ligated into pcDNA3.1 (GenePharma, Shanghai, China) to generate a CPT1A-overexpressing plasmid (Oe-CPT1A). The empty pcDNA3.1 was used as the negative control (Oe-NC). After cell confluence reached 70%, the Oe-CPT1A and Oe-NC plasmids were transfected into HFL-1 cells using Lipofectamine 3000 (Invitrogen) in line with the guidelines. After transfection for 48 h, cells were harvested for subsequent experiments.

### 2.3. Quantitative Real-Time PCR (qRT-PCR)

Total RNA was extracted from cells using a TRIzol reagent (Invitrogen) in line with the manufacturer's instructions. After the reverse transcription from RNA to cDNA using the PrimeScript RT Master Mix Kit (TaKaRa, Japan), qRT-PCR reactions were performed by using the SYBR Premix Ex Taq Kit (TaKaRa, Japan) on a 7500 Fast Real-time PCR System (Applied Biosystems). Ct values were used to calculate the mRNA expression level with *β*-actin as the constitutive marker.

### 2.4. Cell Counting Kit-8 (CCK-8) Assay

Cell viability of HFL-1 cells was determined using the CCK-8 assay. The CCK-8 agent (Dojindo, Japan) was administrated to HFL-1 cells following different treatments. After further incubation at 37°C with 5% CO_2_ for 2 h, the absorbance at 450 nm was detected by a microplate reader.

### 2.5. Enzyme-Linked Immunosorbent Assay (ELISA)

The expression levels of HIF-1*α* (CSB-E12112H), mTOR (CSB-E09038h), TGF-*β*1 (CSB-E04725h), *α*-SMA (CSB-E09343h), and Col-I (CSB-E08082h) in the cell culture media were measured using their corresponding ELISA kits from Cusabio Biotech (Wuhan, China). The expression level of APN in blood and lung tissue homogenate was determined using its ELISA kit (ab108784, Abcam, USA). The level of fatty acid oxidation in cells was detected using its ELISA kit (ab118182). The absorbance at 450 nm was detected by a microplate reader.

### 2.6. Measurement of Lipid Peroxides

The content of malondialdehyde (MDA) was detected by its commercially available kit (A003-1-2) from the Jiancheng Bioengineering Institute (Nanjing, China). The expression level of 4-hydroxy-nonenal (4-HNE) in the cell lysate or tissue lysate was detected using the Lipid Peroxidation (4-HNE) Assay Kit (ab238238, Abcam). The ROS content was detected using its commercial kit (JL13783) from Shanghai Jianglai Biological Technology Co., Ltd. (Shanghai, China).

### 2.7. Immunofluorescence

Treated cells were fixed with 4% paraformaldehyde for 30 min, rinsed with PBS three times for 5 min, and permeated with 0.5% Triton X-100 for 15 min at room temperature. After blockage with 5% BSA for 1 h, cells were incubated with primary antibodies at 4°C overnight. Afterwards, the cells were rinsed with PBS followed by incubation with Alexa Fluor 488-conjugated anti-IgG secondary antibody (ab150077, Abcam) at room temperature for 2 h. The nuclei were stained by DAPI (Vector Laboratories, Inc., USA). The images were observed under a fluorescence microscope (Nikon, Japan).

### 2.8. Western Blot

Total proteins from the cells and lung tissues were extracted with RIPA lysis (Beyotime, Shanghai, China) following instructions. After quantifying the protein concentration using a BCA Protein Assay Kit (Pierce, Rockford, IL), 30 *μ*g/lane of protein was subjected to 15% SDS-PAGE electrophoresis and subsequently transferred onto PVDF membranes. After being blocked with 5% skimmed milk at room temperature for 1 h, the membranes were probed with primary antibodies at 4°C overnight, followed by an incubation with HRP-conjugated secondary antibodies at room temperature for 2 h. Eventually, the immunoreactive bands were developed with the ECL detection system (Amersham Pharmacia Biotech, Amersham, UK) strictly in line with the manufacturer's protocol and quantified using Quantity One software (version 4.6.2; Bio-Rad Laboratories, Inc.).

### 2.9. In Vivo Experiments

Adult female Wistar rats weighing 160~200 g were purchased from the Beijing Vital River Laboratory Animal Technology Co., Ltd. (Beijing, China). All rats were housed under a standard environment with controlled temperature (22 ± 2°C) and humidity (55 ± 5%) and a 12 h/12 h light/dark cycle and allowed free access to food and water. All experimental procedures were approved by the Animal Care Committee of Henan Provincial People's Hospital (Approve No. ZZU-LAC20200911 [6]). The rats were randomly assigned into 5 groups (namely, control, BLM, BLM+C75, BLM+3-MA, and BLM+C75+3-MA, *n* = 6 per group). Rats were treated with a single intratracheal instillation of 5 mg/kg bleomycin (BLM; Nippon Kayaku, Japan) solution to set up an IPF animal model [34]. The rats in the control group received the same volume of the sterilized saline. 14 days after administration of BLM, rats in the other three groups were intraperitoneally injected with 3-methyladenine (3-MA, an autophagy inhibitor, 15 mg/kg; Sigma-Aldrich, USA) and/or intraperitoneally injected with C75 (an agonist of CPT1A, 30 mg/kg; Sigma-Aldrich). On the 21st day, after all rats were anesthetized with 50 mg/kg pentobarbital sodium, the blood was harvested from the abdominal aorta, centrifuged at 4°C for 5 min, and stored at -20°C. The left lung tissue samples were taken out and fixed with 4% paraformaldehyde for histology analysis, while the right lung tissue samples were stored at -80°C for further experiments.

### 2.10. Histology Staining

After fixing with 4% paraformaldehyde for 24 h, the tissue samples were dehydrated in ethanol, embedded in paraffin, cut into 4 *μ*m thick sections, and then stained with haematoxylin and eosin (H&E) solution. The pathological morphology changes were observed under a light microscope (Nikon Microscope, Japan).

### 2.11. Statistical Analysis

Data were expressed as mean ± standard deviation (SD) from at least three independent experiments or groups of 6 rats each. The normal distribution of variables was assessed by the Shapiro-Wilk test. The differences between two groups were determined by Student's *t*-test, and the difference among more than two groups was evaluated by one-way ANOVA analysis, followed by Tukey's post hoc test. A *p* value less than 0.05 was considered to be statistically significant.

## 3. Results

### 3.1. Hypoxia Induces Macrophage M1 Phenotype and Oxidative Stress but Lowers Autophagy and APN/CPT1A Signaling

THP-1 cells were differentiated into M0 macrophages by induction of PMA, followed by hypoxia induction. To explore whether hypoxia could promote macrophage polarization to the M1 subtype, we detected CD86 and iNOS, hallmarks of M1 macrophages. As shown in Figure 1(a), hypoxia induction dramatically elevated the expression level of CD86 and iNOS, suggesting an activation of M1 macrophages upon hypoxia induction. In addition, hypoxia reduced the expression of LC3B, the marked protein of autophagy, indicating a lowered autophagy level caused by hypoxia (Figure 1(b)), which was further confirmed by the reduced protein expression of Beclin-1, Atg5, and LC3B II/I following hypoxia (Figure 1(c)). Meanwhile, hypoxia led to an elevated level of HIF-1*α* and mammalian target of rapamycin (mTOR) (Figure 1(d)). mTOR is a serine/threonine kinase, and the activation of the mTOR pathway can inhibit autophagy [35]. Hypoxia also increased the level of lipid peroxides, such as 4-HNE, MDA, ox-LDL, and ROS (Figure 1(e)). Furthermore, the protein expression of AdipoR1 and CPT1A exhibited a remarkable reduction following hypoxia induction (Figure 1(f)). All the results above verified the changes of macrophage polarization, autophagy, oxidative stress, and fatty acid metabolism following hypoxia.

### 3.2. M1 Macrophages Promote Fibroblast Proliferation and Fibrosis

As hypoxia can induce macrophage polarization to M1 and participate in the progression of pulmonary fibrosis as aforementioned, we would like to explore whether macrophage polarization to M1 plays a critical role during this process and how it functions. A cocultivation system was employed to validate this finding. As shown in Figure 2(a), HFL-1 cells were cultured alone or cocultured with M0/M1 macrophages, and the cell viability of HFL-1 cells cocultured with M0 macrophages exhibited a slight increase, but the cell viability of HFL-1 cells cocultured with M1 macrophages exhibited a remarkable increase, compared to the HFL-1 cells cultured alone. Meanwhile, we also observed a trend towards a higher expression level of TGF-*β*, *α*-SMA, and Collagen I for the M1-treated group (Figures 2(b)–2(d)). The above results possibly suggested the importance of M1 macrophages during fibroblast proliferation and fibrosis.

### 3.3. M1 Macrophages Modulate Fibroblast Autophagy and Fatty Acid Metabolism

As autophagy and fatty acid metabolism were also important factors affected by hypoxia, we subsequently examined the effects of M1 macrophages on autophagy and fatty acid metabolism in HFL-1 cells. As presented in Figure 3(a), in the cocultivation system, the fatty acid oxidation level of HFL-1 cells was obviously suppressed following the coculture with M1 macrophages, which was subsequently verified by the excessive production of lipid peroxides, including MDA and ox-LDL (Figures 3(b) and 3(c)). Afterwards, the downregulated protein expression of AdipoR1 and CPT1A in HFL-1 cells upon the coculture with M1 macrophages revealed that M1 macrophages contributed to a disorder of fatty acid metabolism (Figure 3(d)). In addition, M1 macrophages led to a huge reduction of LC3B-positive HFL-1 cells, as well as the reduced protein expression of Beclin-1, Atg5, and LC3B II/I, revealing a weakened activity autophagy in HFL-1 cells following the coculture with M1 macrophages (Figures 3(e) and 3(f)). The above results demonstrated that M1 macrophages disordered fatty acid metabolism and hindered autophagy in HFL-1 cells.

### 3.4. APN/CPT1A Weakens the Effects of M1 Macrophages on Fibroblast Proliferation, Fibrosis, Autophagy, and Fatty Acid Metabolism

Next, to further explore the regulatory role of fatty acid metabolism during the progression of pulmonary fibrosis, particularly to the induction of macrophages, APN/CPT1A signaling was activated to modulate fatty acid metabolism in HFL-1 cells with the coculture of M1 macrophages. As shown in Figure 4(a), cell transfection was conducted to overexpress CPT1A in HFL-1 cells. Meanwhile, APN (0.5 *μ*g/ml and 2.0 *μ*g/ml) was also introduced to HFL-1 cells. The subsequent western blot assay illustrated that addition of APN or overexpression of CPT1A could greatly elevate the protein expression of AdipoR1 and CPT1A in HFL-1 cells (Figure 4(b)), suggesting that APN/CPT1A signaling was activated. Afterwards, both of APN (2.0 *μ*g/ml) and CPT1A overexpression remarkably lowered HFL-1 cell viability cocultured with M1 macrophages (Figure 4(c)). In addition, APN significantly reduced the levels of TGF-*β*, *α*-SMA, and Collagen I in HFL-1 cells cocultured with M1 macrophages in a concentration-dependent manner, suggesting that APN suppressed M1 macrophage-mediated fibroblast fibrosis. Concurrently, CPT1A overexpression also exerted an antifibrosis activity, and its efficiency was similar to APN (2.0 *μ*g/ml) (Figures 4(d) and 4(e)). Furthermore, APN addition or CPT1A overexpression remarkably elevated the fatty acid oxidation level, reduced the production of MDA and ox-LDL, aggrandized LC3B-positive HFL-1 cells, and improved protein expression of Beclin-1, Atg5, and LC3B II/I in M1 macrophage-mediated HFL-1 cells (Figures 5(a)–5(e)). These above results suggested that activation of APN/CPT1A signaling partly abolished the effects of M1 macrophages on fibroblast proliferation, fibrosis, autophagy, and fatty acid metabolism.

### 3.5. Activation of APN/CPT1A Signaling Alleviates Pulmonary Fibrosis in BLM-Induced IPF Rats

Finally, to validate the critical regulation of APN/CPT1A during the progression of IPF, we successfully established an IPF rat model using BLM injection. In addition, the BLM-induced rats were injected with C75 and/or 3-MA for treatment. The histological analysis presented in Figure 6(a) illustrated that the injured pulmonary tissues in IPF rats were greatly improved by C75 treatment, but this protection by C75 was partly weakened when rats were treated with both C75 and 3-MA. The following western blot assay exhibited that BLM caused a huge rise of the protein expression level of TGF-*β*, *α*-SMA, and Collagen I in pulmonary tissues, whereas C75 treatment lowered this rise, indicating that C75 protected rats against fibrosis; however, this antifibrosis effect of C75 was then partly weakened by the simultaneous treatment of 3-MA (Figure 6(b)). In addition, the lipid peroxides including 4-HNE, MDA, and ox-LDL in pulmonary tissues were obviously increased by BLM induction but were reduced following C75 treatment. 3-MA treatment alone had no influence on lipid peroxides, but cotreatment with 3-MA and C75 led to the elevation of lipid peroxides again compared to C75 treatment alone in BLM-induced rats (Figures 6(c)–6(e)). What is more, it was observed that the APN level in blood or pulmonary tissue was reduced following BLM stimulation, which was reversed by C75 treatment, and the effect of C75 was partly weakened by additional 3-MA treatment (Figures 6(f) and 6(g)). The following protein expression of AdipoR1 and CPT1A in pulmonary tissues exhibited a similar trend to the APN level following different treatments (Figure 6(h)). Furthermore, the BLM-induced IPF rat presented as a low activity of autophagy, evidenced by the downregulated protein expression of Beclin-1, Atg5, and LC3B II/I. C75 treatment obviously promoted the activation of autophagy of IPF rats, which was partly hindered by 3-MA (Figure 6(i)). Taken together, these results suggested that activation of APN/CPT1A signaling effectively alleviated fibrosis and excessive fatty acid oxidation in BLM-induced rats, which was partly abolished when autophagy was inhibited.

## 4. Discussion

IPF is a chronic progressive interstitial lung disease that leads rapidly to death. The incidence of pulmonary fibrosis keeps increasing and brings great burden to global healthcare. Thus, exploring the pathogenesis of IPF and discovering novel effective targets for IPF treatment are essential. Currently, accumulating evidence discloses that the alternations of fatty acid metabolism are commonly detected in fibrosis diseases. In the present study, we uncovered a critical function for APN/CPT1A-mediated lipid acid metabolism in the development of pulmonary fibrosis. Here, we disclosed that hypoxia induced macrophage polarization to M1, which was beneficial to fibroblast proliferation and fibrosis formation *in vitro*, accompanied with a disorder of the APN/CPT1A pathway which is critical for lipid acid metabolism, an overproduction of lipid peroxides, and an activation of autophagy. Thereafter, APN treatment or CPT1A overexpression greatly suppressed lipid peroxide accumulation, fibroblast proliferation, and profibrotic protein expression but activated autophagy *in vitro*. The following *in vivo* experiments further validated the protection of CPT1A overexpression in pulmonary fibrosis; however, the antifibrosis property of CPT1A was partly abolished by 3-MA, indicating that APN/CPT1A-mediated fatty acid metabolism exerted its protective role in IPF partly through activating autophagy.

Fibroblasts are effector cells driving the progress of fibrotic diseases including IPF featured as unrestrained deposition and stiffening of the extracellular matrix. Despite diverse and varied etiologies of fibrotic diseases, it is pointed out that macrophages play a critical role in the initiation and development of fibrosis [36]. Macrophages can influence fibroblasts through direct cell-cell interactions or via indirect signals [37]. For instance, Bhattacharya and colleagues found that activated macrophages could promote fibroblast proliferation and migration in vitro through the expression of platelet-derived growth factor (PDGF) and TGF-*β* [38]. In addition, selective depletion of interstitial macrophages could limit lung fibrosis in response to BLM *in vivo* [39]. Thus, macrophage-fibroblast crosstalk acts as a crucial pathway for the initiation and development of IPF. It is well known that hypoxia is an important microenvironmental factor in the development of tissue fibrosis. Here, macrophages were polarized to M1 macrophages following hypoxia induction, which were then cocultured with HFL-1 cells. As expected, M1 macrophages improved the cell viability of HFL-1 cells and promoted the expression level of TGF-*β*, *α*-SMA, and Collagen I, revealing that hypoxia induced the generation of M1 macrophages, which subsequently promoted the fibroblast proliferation and fibrosis. Nevertheless, in this study, in addition to verifying the influences of macrophages on fibroblast proliferation and fibrosis, more attention was focused on the influences on autophagy, oxidative stress, and fatty acid metabolism following hypoxia.

Emerging evidence uncovered that alterations in fatty acid metabolism are core pathways and common mechanisms which play a crucial role in multiple fibrotic disorders, including kidney fibrosis, liver fibrosis, and pulmonary fibrosis [40]. Excessive accumulation of lipid induces cellular lipotoxicity potentially contributing to fibrosis progression [41]. Thus, alterations in fatty acid metabolism through gene variation or pharmacological targeting of lipid metabolic processes may be an alternative strategy to inhibit fibrosis development. In pathological conditions, the lipid peroxides accumulate and affect cell viability and function. Elevated levels of lipid peroxides, such as 4-HNE, or their protein adducts have been evidenced in lung tissues and bronchoalveolar fluids in patients suffering from IPF [42, 43]. The excessive production of lipid peroxides can directly cause oxidative stress, which will arouse or even sharpen the inflammatory injuries, resulting in body damage. Recently, it is observed that the increase or the reduction of oxidative stress markers is independent of different biological specimens of patients with IPF, highlighting the proposition that oxidative stress is one of the most relevant pathophysiological mechanisms involved in IPF [43, 44]. Oxidative stress will lead to alternations in the tissue microenvironment favoring fibrosis and stimulate myofibroblast differentiation and collagen deposition, contributing to a profibrotic event [3]. Consistently, in this study, we not only found excessive accumulation of 4-NHE, MDA, and ox-LDL in pulmonary fibrosis *in vitro* and *in vivo*, accompanied with the elevated expression of profibrotic proteins, including TGF-*β*, *α*-SMA, and Collagen I, but also demonstrated that strengthening of APN/CPT1A signaling was beneficial to restore the balance of lipid peroxides and profibrotic proteins, so as to suppress oxidative stress and alleviate pulmonary fibrosis.

Last, but not least, fatty acid metabolism is closely associated with autophagy. It has been proposed that cells may be unable to deal with lipid droplets via acid lipases in the absence of autophagy, leading to the reduction of mitochondrial *β*-oxidation and accumulation of excessive lipids, suggesting that fatty acid oxidation may be mediated through an autophagy-dependent mechanism [45, 46]. Coincidently, it is reported that APN can regulate the activation of autophagy *in vivo* and *in vitro*, and APN exerts as a novel therapeutic target of diabetic retinopathy through inhibiting autophagy [47]; however, APN exhibits a protective role against Alzheimer-like pathologies via triggering autophagy [48], emphasizing a dual relationship between APN and autophagy in different diseases. In fibrotic diseases, Li et al. found that APN attenuated hypertension-induced renal fibrosis via promoting epithelial autophagy [49]; Qi et al. reported that APN suppressed angiotensin II-induced cardiac fibrosis through activating macrophage autophagy [30]. Consistently, in this study, we also found an activation of autophagy upon APN treatment in M1 macrophage-induced HFL-1 cells, evidenced by elevated LC3-positive cells and upregulated protein expressions of Beclin-1 and Atg5, confirming that APN might attenuate fibrotic diseases through activating autophagy. Furthermore, CPT1A overexpression exerts similar effects on the autophagy level in comparison to APN in M1 macrophage-induced HFL-1 cells. Furthermore, the protective role of CPT1A overexpression against oxidative stress, lipid peroxide overproduction, and fibrosis in BLM-induced IPF rats was partly hindered by simultaneous treatment of 3-MA. Given that the APN/CPT1A pathway is critical to fatty acid metabolism that is also closely associated with autophagy, the activation of autophagy may partly explain the protection of APN/CPT1A-mediated fatty acid metabolism in IPF.

## 5. Conclusion

In summary, we demonstrated not only that hypoxia-induced macrophage polarization to M1 could induce pulmonary fibrosis but also that the activation of APN/CPT1A-mediated fatty acid metabolism suppressed lipid peroxide accumulation and fibroblast proliferation but activated autophagy in IPF. Mechanically speaking, the protective role of APN/CPT1A-mediated fatty acid metabolism was autophagy-dependent. Therefore, targeting fatty acid metabolism is an effective approach for the treatment of IPF.

## Figures and Tables

**Figure 1:** Hypoxia induces macrophage M1 phenotype and oxidative stress but lowers autophagy and APN/CPT1A signaling. THP-1 cells were differentiated into M0 macrophages by induction of PMA, followed by hypoxia induction. (a) The level of CD86 and iNOS was detected by immunofluorescence. (b) The LC3B-positive cells were determined using immunofluorescence and observed under a fluorescence microscope. (c) The protein expression of beclin-1, Atg5, and LC3B II/I was measured by western blot. (d) The level of HIF-1*α* and mTOR was detected by ELISA. (e) The level of lipid peroxides, such as 4-HNE, MDA, ox-LDL, and ROS, was measured using their commercial kits, respectively. (f) The protein expression of AdipoR1 and CPT1A was measured using western blot. ^∗∗∗^*p* < 0.001 vs. M0.

**Figure 2:** M1 macrophages promote fibroblast proliferation and fibrosis. HFL-1 cells were cultured alone or cocultured with M0/M1 macrophages. (a) The cell viability of HFL-1 cells was detected by CCK-8 assay. ^∗∗∗^*p* < 0.001 vs. HFL-1. The level of (b) TGF-*β*, (c) *α*-SMA, and (d) Collagen I in HFL-1 cells was detected using their corresponding ELISA kits. ^∗∗∗^*p* < 0.001 vs. blank.

**Figure 3:** M1 macrophages modulate fibroblast autophagy and fatty acid metabolism. HFL-1 cells were cultured alone or cocultured with M0/M1 macrophages. (a) The fatty acid oxidation level of HFL-1 cells was detected by its ELISA kit. (b) The MDA level of HFL-1 cells was detected by its commercial kit. (c) The ox-LDL level of HFL-1 cells was detected by its commercial kit. (d) The protein expression of AdipoR and CPT1A in HFL-1 cells was detected using western blot. (e) The LC3B-positive cells were determined using immunofluorescence and observed under a fluorescence microscope. (f) The protein expression of Beclin-1, Atg5, and LC3B II/I in HFL-1 cells was detected using western blot. ^∗^*p* < 0.05 and ^∗∗∗^*p* < 0.001 vs. blank.

**Figure 4:** APN/CPT weakens the effects of M1 macrophages on fibroblast proliferation and fibrosis. (a) HFL-1 cells were transfected with Oe-NC or Oe-CPT1A, and the mRNA level of CPT1A was measured by qRT-PCR. ^∗∗∗^*p* < 0.001 vs. Oe-NC. (b) Cell transfection was conducted to overexpress CPT1A in HFL-1 cells. Meanwhile, APN (0.5 *μ*g/ml and 2.0 *μ*g/ml) was introduced to HFL-1 cells. HFL-1 cells were cocultured with M1 macrophages. The protein expression of AdipoR and CPT1A in HFL-1 cells was detected using western blot. (c) The cell viability of HFL-1 cells was detected by CCK-8 assay. The level of (d) TGF-*β*, (e) *α*-SMA, and (f) Collagen I in HFL-1 cells was detected using their corresponding ELISA kits. ^∗^*p* < 0.05 and ^∗∗∗^*p* < 0.001 vs. HFL-1+M1; ^##^*p* < 0.01 and ^###^*p* < 0.001 vs. HFL-1+M1+Oe-NC.

**Figure 5:** APN/CPT1A weakens the effects of M1 macrophages on fibroblast autophagy and fatty acid metabolism. Cell transfection was conducted to overexpress CPT1A in HFL-1 cells. Meanwhile, APN (0.5 *μ*g/ml and 2.0 *μ*g/ml) was introduced to HFL-1 cells. HFL-1 cells were cocultured with M1 macrophages. (a) The fatty acid oxidation level of HFL-1 cells was detected by its ELISA kit. (b) The MDA level of HFL-1 cells was detected by its commercial kit. (c) The ox-LDL level of HFL-1 cells was detected by its commercial kit. (d) The LC3B-positive cells were determined using immunofluorescence and observed under a fluorescence microscope. (e) The protein expression of Beclin-1, Atg5, and LC3B II/I in HFL-1 cells was detected using western blot. ^∗∗^*p* < 0.01 and ^∗∗∗^*p* < 0.001 vs. HFL-1+M1; ^###^*p* < 0.001 vs. HFL-1+M1+Oe-NC.

**Figure 6:** Activation of APN/CPT signaling alleviates pulmonary fibrosis in BLM-induced IPF rats. An IPF rat model was established by injection of BLM, and the BLM-induced rats were injected with C75 and/or 3-MA for treatment. (a) The histological analysis was conducted by H&E staining. (b) The protein expression level of TGF-*β*, *α*-SMA, and Collagen I in pulmonary tissues was measured using western blot. (c–e) The levels of the lipid peroxides including 4-HNE, MDA, and ox-LDL in pulmonary tissues were detected using their commercial kits, respectively. The level of APN (f) in blood and (g) in pulmonary tissue was measured by ELISA. (h) The protein expression of AdipoR1 and CPT1A in pulmonary tissues was detected by western blot. (i) The protein expression of Beclin-1, Atg5, and LC3B II/I in pulmonary tissues was detected by western blot. ^∗∗∗^*p* < 0.001 vs. blank; ^#^*p* < 0.05, ^##^*p* < 0.01, and ^###^*p* < 0.001 vs. BLM; ^+^*p* < 0.05, ^++^*p* < 0.01, and ^+++^*p* < 0.001 vs. BLM+C75.

## Data Availability

All data generated in this study have been included in this article.
